The article "A Model of Spatial Cell Development in Rat Hippocampus Based on Artificial Neural Network" was retracted in 2023. Reasons: signs of a paper mill; compromised peer review; unreliable results or conclusions.

# A Model of Spatial Cell Development in Rat Hippocampus Based on Artificial Neural Network

**DOI:** 10.1155/2021/5607999

**Published:** 2021-10-26

**Authors:** Naigong Yu, Hejie Yu, Yishen Liao, Zongxia Wang, Ouattara Sie

**Affiliations:** Faculty of Information Technology, Beijing University of Technology, Beijing Key Laboratory of Computational Intelligence and Intelligent System, Beijing 100124, China

## Abstract

Physiological studies have shown that the hippocampal structure of rats develops at different stages, in which the place cells continue to develop during the whole juvenile period of rats and mature after the juvenile period. As the main information source of place cells, grid cells should mature earlier than place cells. In order to make better use of the biological information exhibited by the rat brain hippocampus in the environment, we propose a position cognition model based on the spatial cell development mechanism of rat hippocampus. The model uses a recurrent neural network with parametric bias (RNNPB) to simulate changes in the discharge characteristics during the development of a single stripe cell. The oscillatory interference mechanism is able to fuse the developing stripe waves, thus indirectly simulating the developmental process of the grid cells. The output of the grid cells is then used as the information input of the place cells, whose development process is simulated by BP neural network. After the place cells matured, the position matrix generated by the place cell group was used to realize the position cognition of rats in a given spatial region. The experimental results show that this model can simulate the development process of grid cells and place cells, and it can realize high precision positioning in the given space area. Moreover, the experimental effect of cognitive map construction using this model is basically consistent with the effect of RatSLAM, which verifies the validity and accuracy of the model.

## 1. Introduction

In the adult rat brain, space and orientation are expressed by the hippocampal structure, which is home to a variety of spatial cells with specific firing effects on spatial location, including head-direction cells [1], grid cells [2], and place cells [3]. Each spatial cell receives the motion information of the body or the outside world [4, 5], and processing and handling this information form a cognitive map based on the current spatial environment in the hippocampus structure [6, 7]. In 1971, O'Keefe et al. found a cell that is selective for spatial location in the hippocampus structure of the rat brain [8]. The characteristic of this cell is that only when the rat is in a specific position in space, it will discharge activity, so it is called a place cell, and the space corresponding to its discharge is called a place cell discharge field (abbreviated as place field) [9]. The place cell establishes the mapping relationship between the brain area and the external physical world [10], and it is the basis of the cognitive map [11]. In 2005, Hafting et al. found another neuronal cell in the entorhinal cortex of rats that has a strong discharge characteristic for spatial location through related experiments; it will produce periodic discharges in a specific area in space [12, 13]. Different from the firing rules of place cells, the firing field of this cell is in the form of a regular hexagon throughout the entire spatial area. This kind of neuron cell that also has firing characteristics for the spatial position is called a grid cell [14, 15], and the spatial area corresponding to its discharge is called the grid cell discharge field (referred to as the grid field).

This leads to a question as to whether the ability of each spatial cell in the hippocampus structure to show its specific discharge to space is innate, or with the gradual growth of rats, each spatial cell can gradually show the above-mentioned discharge characteristics. Physiological studies have shown that the cells in the hippocampus structure of the rat brain develop and mature at different stages. A study by Wills et al. in 2010 revealed the presence of multiple spatial neuronal representations in the hippocampal structures of the rat brain and showed how they develop with age. Among them, the discharge characteristics of the grid cells gradually mature in about 3-4 weeks after the rat's eyes are opened, and the place cells continue to develop throughout the juvenile period of the rat and reach maturity after the juvenile period [16]. The development process of grid cells and place cells recorded by electrophysiology is shown in Figure 1. The discharge characteristics of the two types of neurons gradually mature and stabilize with age.

Exploring the cognitive mechanism of the brain and assigning this mechanism to an artificial system or machine constitute a topic of common concern to artificial intelligence and robotics, as well as neurophysiology and psychology. Rodents (rats are often used as experimental objects in biological experiments) have been used as biological experimental research objects for more than a century. Not only their behavioral and psychological manifestations have been extensively studied, but their brain anatomical structure and neurophysiological operating mechanism have been also researched in depth. In recent years, based on the anatomical structure of the rat brain and the mechanism of environmental cognition, there has been endless research on the construction of a rodent-like brain model of environmental cognition [17–19]. At this stage, there are two main aspects of robot navigation research based on the cognitive mechanism of the rat brain hippocampus environment. One is to build a neural network model based on the anatomical structure of the hippocampus and the cognitive mechanism of spatial cells and apply it to mobile robots that mimic the rat brain nervous system for autonomous navigation [20]. The other is robot real-time localization and map construction based on rat brain hippocampus neuroethology [21].

Fast and accurate positioning of oneself in the environment has always been an important task in the field of intelligent mobile robots. The “RatSLAM” framework has obtained extensive and in-depth research on the cognitive computational neurobehavioral model of the rat brain hippocampus environment and proposed a mature real-time positioning and map construction method, whose core part is called the pose cell [22, 23]. Since pose cells are not spatial cells in the hippocampus structure of the rat brain, the algorithm mainly mimics the neurobehavioral characteristics of rats, rather than being completely based on the anatomical and physiological characteristics of the hippocampus structure. In 2014, Hasselmo Lab proposed an algorithm that combines a hierarchical forward predictive trajectory model with the RatSLAM model [24]. The specific process is to use the RatSLAM model to transform spatial information into visual spatial experience maps in a visualized external environment, so that the robot can conduct autonomous navigation in the outdoors more humanely. However, the lack of feedback loop of this model makes it not particularly good in large-scale physical navigation. In this period, most research on the mechanism of imitation of the hippocampus mainly focused on spatial cell modeling [25] and hippocampal circuit information transmission modeling [26]. However, there is relatively little research on the development of various spatial cells.

Therefore, we propose a spatial cognition model based on the developmental mechanism of spatial cells in the hippocampus of the rat. This model uses a unified computer system to simulate the changes in the discharge characteristics of grid cells and place cells during development and combines the discharge characteristics of place cells to achieve accurate expression of the rat position in the active area. This article has made progress in the following two aspects: 1. In public studies, this model is the first to use neural networks to simulate the changes in discharge characteristics during the development of two spatial cells (grid cell and place cell) in the rat brain hippocampus structure. 2. Compared with the positioning method of traditional mobile robots, the position recognition model is more bionic and suitable (low requirements on hardware and sensors) for navigation in different environments.

## 2. Materials and Methods

### 2.1. The Overall Structure of the Model

This section explains in detail the overall structure and principle of the positional cognitive model based on the developmental mechanism of the rat brain hippocampus spatial cells. It is mainly divided into the following three aspects: (1) This article uses RNNPB to simulate the changes in discharge characteristics during the development of fringe cells and then indirectly simulates the development of grid cells through the fusion of fringe waves in three directions through the oscillatory interference mechanism. (2) The output of the grid cell is used as the information input of the place cell, and the BP neural network is used to simulate the development process of the place cell. (3) After the place cells have matured, the place matrix generated by the place cell group can be used to realize the rat's location cognition in the space. The overall operating mechanism of the model is shown in Figure 2.

### 2.2. Grid Cell Development Process

Many studies have shown that the stripe cells in the superficial area of the proximal parenchyma and the entorhinal cortex are a cell group with periodic stipe-like discharge fields on a two-dimensional plane [27]. The striped wave is the necessary input information for the grid field generation. Its essence is that a two-dimensional cos wave generated by the three 60° oriented stripe cell families can form a regular hexagonal grid wild arrangement throughout the entire space through the theory of oscillation interference [28–30]. The mechanism of the stripe wave generating the regular hexagonal discharge field of the grid cell is shown in Figure 3.

In the oscillating interference model, the main driving signal for the stripe cells to produce striped waves is the self-motion clue information of the rat. The recurrent neural network with parametric bias (RNNPB) model was proposed by Tina [31]. It can simulate the process of cognitive development on the agent, so it is widely used in the modeling of cognitive development. Therefore, we use RNNPB to simulate the development of a single stripe cell. Then, the fringe waves in three directions are merged through the oscillation interference mechanism to indirectly simulate the grid cell development process. The development mechanism of the grid field based on RNNPB is shown in Figure 4.

The RNNPB model is essentially a predictor in the simulation of spatial cell development in intelligences. It consists of a three-layer structure (input, hidden, and output layers) with cyclic feedback from the output layer to the input layer. Therefore, it has a network parameter *ψ* consisting of two weight matrices and two bias vectors: *ψ* = {*w*_21_, *w*_32_, *b*_1_, *b*_2_}. We mainly use its learning and prediction modes to model changes in discharge properties during stripe cell development. In the learning mode, the input is the current state *S*(*t*) and the bias parameter PB, and the output is the next state *S*(*t*+1). *S*(*t*) and *S*(*t*+1) represent the discharge rate of the stripe cell at the current moment and the next moment. The PB node represents the magnitude of the velocity component of the self-moving velocity in the direction of the striped wave. The RNNPB structure in the learning mode is shown in Figure 5(a). The model uses the prediction difference to calculate and correct the connection weight of the neural network in real time through the BPTT algorithm [32]. Combined with the learning of the PB node, the RNNPB model autonomously realizes the mapping relationship between the PB value and the time series.

The main role of the RNNPB is to generate memory in the form of a time series of stripe cell discharge rates. Therefore, the PB units have static values *c* as an input when the discharge memory is formed, whereas the values of the context units change for each time step based on the recurrent connection from the context output unit of the context input unit of the current time step *X*(*t*) to the context input unit of the next time step *X*(*t*+1). The hidden unit values at the *t *+* *1-th time step *H*(*t*+1) are produced with weight *w*_21_ and bias *b*_1_ from the input unit values at the current time step *S*(*t*), the PB values *c*, and the context unit values at the current time step *X*(*t*) as shown in (1). The output unit values *S*(*t*+1) and the context output values *X*(*t*+1) at the *t*+1-th time step are produced with weight *w*_32_ and bias *b*_2_ from the hidden unit values as shown in (2).

(1) $$\begin{array}{c} H\left(t+1\right)=\text{sigmoid}\left(w_{21}•\left[\begin{array}{c} S\left(t\right)\\ c\\ X\left(t\right) \end{array}\right]+b_{1}\right), \end{array}$$

(2) $$\begin{array}{c} \left[\begin{array}{c} S\left(t+1\right)\\ X\left(t+1\right) \end{array}\right]=\text{sigmoid}\left(w_{32}•H\left(t\right)+b_{2}\right). \end{array}$$

The values of the BP bias parameters used for learning in this paper are the input velocity and angle information; the length of the sequence is denoted by *L*. In the output of each learning model, the error about the PB node is fed back for calculation and used in the calculation of the neural network connection weights, and the BPTT algorithm is used to determine the optimal network parameters. Similar to the back-propagation algorithm in feedforward neural networks, the error *E*_out_(*t*+1) between a generated stripe cell discharge rate *S*_gen_(*t*+1) and a given stripe cell discharge rate *S*_ref_(*t*+1) at the *t *+* *1-th time step is back-propagated from the third layer to the first layer. When the length of the desired time series is *L*, the recurrent connections of the context units are unfolded through time, and the unfolded network is then identical to a deep feedforward neural network that has 3*L* layers. The network parameter *ψ* is updated iteratively through back-propagation as follows:

(3) $$\begin{array}{c} \Delta w_{32,ij}=\varepsilon \sum_{n=1}^{L}H_{n,j}\left\{\begin{array}{cc} \delta_{\text{out},n,i}, & \text{if }i\in \text{output unit},\\ \delta_{cxt,n,i}, & \text{if }i\in \text{context unit}, \end{array}\right. \end{array}$$

(4) $$\begin{array}{c} \Delta b_{3,i}=\sum_{n=1}^{L}\left\{\begin{array}{cc} \delta_{\text{out},n,i}, & \text{if }i\in \text{output unit},\\ \delta_{cxt,n,i}, & \text{if }i\in \text{context unit}, \end{array}\right. \end{array}$$

(5) $$\begin{array}{c} \Delta w_{21,ij}=\varepsilon \sum_{n=1}^{L}\delta_{\text{hid},n,i}\left\{\begin{array}{cc} S_{n-1,j}, & \text{if }j\in \text{output unit,}\\ c_{n,j}\text{,} & \text{if }j\in PB\text{ unit,}\\ X_{n-1,j}, & \text{if }i\in \text{context unit,} \end{array}\right. \end{array}$$

(6) $$\begin{array}{c} \Delta b_{2,i}=\varepsilon \sum_{n=1}^{L}\delta_{\text{hid},n,i}, \end{array}$$

(7) $$\begin{array}{c} \Delta X=k_{bp}\sum_{n=1}^{L}\delta_{\text{PB},n}. \end{array}$$

Through these sequential learning, the RNNPB model produces a series of outputs corresponding to the PB values of the inputs, thus modeling the changes in discharge characteristics during the development of the stripe cells and establishing the relationship between the discharge rate of the grid cells and the self-motion cues in a given spatial region. The learning process determines the magnitude of the connection weights in the recurrent neural network, at which point the output nodes in the open-loop prediction approach in Figure 5(a) are joined to the input nodes to form the closed-loop network structure shown in Figure 5(b). Thus, in the closed-loop mode, the output of the next time step is fed back to the current step input, allowing prediction of the size of the stripe cell discharge rate for any future step.

After the corresponding firing activation sequence of the stripe cell is obtained, the corresponding firing activation sequence of the grid cell can be obtained through the oscillation interference mechanism. If the discharge rate sequence of the stripe cell is *S*_(*i*, *j*)_(*t*), the mathematical expression of the discharge rate *g*_*j*_(*t*) of the *j*-th grid cell is shown in.

(8) $$\begin{array}{c} g_{j}\left(t\right)=\sum_{i=1}^{3}S_{\left(i,j\right)}\left(t\right). \end{array}$$

In (8), j is the number of the grid cells and i is the number of the stripe cells that generate the *j*-th grid cell grid field, where the value of *i* is 1∼3, respectively, representing the stripe wave direction *α* + 60°, *α* + 120°, and *α* + 180° stripe cells. With the BPTT time back-propagation error and the learning of PB nodes, the RNNPB connection weights are continuously updated and corrected, and the firing rate *g*_*j*_(*t*) can gradually approach the regular hexagonal firing field, thereby simulating the grid cell development process.

### 2.3. Place Cell Development Process

The place cell is a kind of discharge cell that is selective to the spatial location. Only when the rat is in a specific position in the space, the cell will discharge activity. We used the place cell mathematical model provided by O'Keefe et al. [33] to calculate the discharge rate of the place cell at the current position, and its mathematical expression is shown in.

(9) $$\begin{array}{c} R_{pc}^{i}\left(r\right)=\exp\left(-\frac{{\left\|r-r_{i0}\right\|}^{2}}{\sigma^{2}}\right). \end{array}$$

In (9), *R*_*pc*_^*i*^(*r*) is the discharge rate of the place cell at the position *r*, *r*=[*x*, *y*] represents the current position coordinates of the rat in the environment; *r*_*i*0_ is the position coordinate corresponding to the center of the firing field of the place cell; and *σ*^2^ is the adjustment coefficient of the firing field of the place cell.

The forward input of the place cell is the output of the grid cell, and the grid cells of different scales are discharged into the place cell [34]. Based on this, the BP feedforward neural network is designed to simulate the firing activation characteristics during the development of place cells. The neural network structure is shown in Figure 6. Using BP neural network to simulate the changes of discharge characteristics during the development of place cells mainly includes the following steps: 1. obtaining a sample set of place cell development; 2. using BP neural network to realize the process of mapping from grid cells to place cells; 3. testing the developmental maturity of the place cell discharge activation characteristics.

**Step 1 .**

Place cell development sample

The input of the BP neural network developed by the place cells is the set of firing rates of the grid cell population at the current time and the previous time, and the output is the set of firing rates of the place cell population. To facilitate calculations and obtain more accurate discharge rate effects, we represent all input and output nodes in the BP neural network with binary numbers; that is, 0 and 1 are the resting state and the excited state of the cell discharge activity, respectively. Suppose that the discharge rate function of the *j*-th grid cell and the *i*-th place cell at time *t* after binarization is as follows:

(10) $$\begin{array}{c} gm_{\left(j\right)}\left(t\right)=\left\{\begin{array}{cc} 1, & \left(t\right)>TH_{gc},\\ 0, & g_{i}\left(t\right)<TH_{gc}, \end{array}\right. \end{array}$$

(11) $$\begin{array}{c} pm_{\left(i\right)}\left(t\right)=\left\{\begin{array}{cc} 1, & R_{pc}^{i}\left(r\right)>TH_{pc},\\ 0, & R_{pc}^{i}\left(r\right)<TH_{pc}. \end{array}\right. \end{array}$$

Among them, *TH*_*gc*_ and *TH*_*pc*_, respectively, represent the set thresholds for binarization of firing rate of grid cells and place cells. Based on this, a place cell development sample set with grid cell firing rate as input and place cell firing rate as output can be established.

**Step 2 .**

Development process

After establishing the place cell development sample set, it is necessary to use the training data to train the neural network. Considering the rapidity and accuracy of the place cell development process, we use the Levenberg–Marquardt BP algorithm [35] with faster iterative convergence speed to simulate the development process of the place cell's single discharge characteristics. In the specific training process, to prevent the neural network from falling into a local minimum state, we initialize the BP neural network connecting the grid cells and the place cells with multiple sets of different parameter values and take the solution with the smallest error after training as the final parameter to improve the accuracy and generalization of the model. Through the training of the neural network, the output of the neural network gradually shows the discharge characteristics of a single place field of the place cell. After the development is completed, the output of the neural network is *pc*_(*i*)_^develop^(*t*), which is the set of the place cell firing rate with the movement of the rat.

**Step 3 .**

Developmental maturity test

In Wills' experiment, the method for testing the maturity of place cells is to count the 95% discharge accuracy standards for each time, which corresponds to the proportion of 95% of the spatial response accuracy of cells in all locations under the time node. Therefore, the method for judging the developmental maturity of the discharge characteristics of the place cells used in this article is to use the place cell firing rate binarization threshold *TH*_*pc*_ and the place cell firing rate formula (9). Then, the radius of the cell discharge field area at the *i*-th position can be obtained as follows:

(12) $$\begin{array}{c} {\text{Rad}}_{i}=\sqrt{-\sigma^{2}\ln\left(TH_{pc}\right)}. \end{array}$$

As shown in Figure 7, the green circle is the cell discharge field area with a radius of Rad_*i*_. The red discharge point is inside the circle, which represents a correct discharge response; the black discharge point is outside the circle, which represents a wrong discharge response.

### 2.4. Positioning Model

Place cells are the main source of information for rats to know where they are in the environment. We propose an iterative method for the position matrix. The specific process is that in a given space area, when the agent appears in a certain position in space, place cells in different positions can show different discharge effects. Therefore, using the discharge activity of place cells in multiple locations in this area as an iterative sample for iterative calculations, the agent can accurately locate its own position in the environment. On this basis, the judgment of the convergence of the position matrix is added in the calculation process of the iterative model, and the number of iterations is dynamically adjusted to improve the accuracy and efficiency of the model. The operation mechanism of the iterative model using place cells for positioning is shown in Figure 8.

It is known that the firing rate of the *i*-th place cell obtained by the developmental model at time *t* is *pc*_(*i*)_^develop^(*t*). To make the place cell show the position of the agent, suppose that the iterative matrix of the *i*-th position cell at time *t* is mat_(*m*, *n*)_^placecell_*i*_^(*t*). If the conversion ratio between the iterative matrix and the real environment is *β*, the length and width of the rectangular area of the real environment covered by the iterative matrix are (*β*_*m*_, *β*_*n*_). The mathematical expression for solving the iterative matrix of place cells is.

(13) $$\begin{array}{c} {\text{mat}}_{\left(m,n\right)}^{{\text{placecell}}_{i}}\left(t\right)=\left\{\begin{array}{c} \left\{\begin{array}{cc} 1 & \sqrt{{\left(\beta m-x_{i0}\right)}^{2}+{\left(\beta n-y_{i0}\right)}^{2}}<{\text{Rad}}_{i}\\ 0 & \sqrt{{\left(\beta m-x_{i0}\right)}^{2}+{\left(\beta n-y_{i0}\right)}^{2}}>{\text{Rad}}_{i} \end{array},pc_{\left(i\right)}^{\text{develop}}\left(t\right)>TH_{pc},\right.\\ \left\{\begin{array}{cc} 0 & \sqrt{{\left(\beta m-x_{i0}\right)}^{2}+{\left(\beta n-y_{i0}\right)}^{2}}<{\text{Rad}}_{i}\\ 1 & \sqrt{{\left(\beta m-x_{i0}\right)}^{2}+{\left(\beta n-y_{i0}\right)}^{2}}>{\text{Rad}}_{i} \end{array}\right.,pc_{\left(i\right)}^{\text{develop}}\left(t\right)<TH_{pc}. \end{array}\right. \end{array}$$

In (13), *r*_*i*0_=[*x*_*i*0_, *y*_*i*0_] represents the center coordinates of the firing field of the cell at the *i*-th position, and Rad_*i*_ is the radius of the firing field of the cell at the *i*-th position.

Suppose that the matrix storing the position information of the agent at time *t* is the position matrix mat_(*m*, *n*)_^placecell_*i*_^(*t*). The number of rows and columns *m*, *n* and the area covered are the same as the number of rows and columns of the iterative matrix. The meaning of the position matrix is as follows: a matrix element of 1 means that the agent may be in the current position, and a matrix element of 0 means that the agent is unlikely to be in the current position. For the position matrix to accurately express the current position of the agent, it is required that the elements of 1 in the position matrix are sufficiently small and sufficiently concentrated. Therefore, it is necessary to use multiple iterative matrices corresponding to multiple place cells to iteratively solve the position matrix. The number expression is as follows:

(14) $$\begin{array}{c} {\text{mat}}_{\left(m,n\right)}^{\text{position}}\left(\text{t}\right){=\text{mat}}_{\left(m,n\right)}^{\text{position}}\left(\text{t}\right).*\;{\text{mat}}_{\left(m,n\right)}^{{\text{placecell}}_{i}}\left(\text{t}\right). \end{array}$$

In (14),*∗* represents the bitwise sum of the elements of the corresponding rows and columns of the matrix.

In this way, after each iterative operation, the iterative matrix will transfer the position information of the agent it carries to the position matrix. With the increase of the number of iterations, the possible positions of the agent on the position matrix gradually decrease, which means that the position of the agent is gradually clear. When the number of iterations is enough, the position matrix will be able to accurately express the current position of the agent.

When using the iterative matrix to solve the position matrix, if the number of iterations is constant, the position matrix may have enough accurate information to express the position of the agent before the iteration is completed. Therefore, the fixed number of iterations is not conducive to the efficiency of the algorithm. We adopt a method of calculating the convergence of the position matrix to determine whether the position matrix can get enough accurate information to express the position of the agent, to determine whether to continue the iteration. The specific procedure is as follows: traverse the position matrix, retrieve all elements of 1 in the matrix, and count their corresponding horizontal and vertical coordinates into two sets of coordinate sequences *x*_coor_ and *y*_coor_. Next, respectively, solve the variances of the two sets of sequences as Var(*x*_coor_) and Var(*y*_coor_).

Setting a judgment threshold *TH*_detection_, when Var(*x*_coor_) < *TH*_detection_ and Var(*y*_coor_) < *TH*_detection_are satisfied at the same time, it is judged that the position matrix has converged enough to accurately express the information of the agent's position and the iteration is stopped; otherwise, continue to execute the iteration. After a sufficiently convergent position matrix is obtained, the current position of the agent needs to be obtained through the information of the position matrix. The specific method is as follows: also take the two sets of coordinate sequences *x*_coor_ and *y*_coor_ that are 1-element horizontal and vertical coordinate statistics in the position matrix. Let *num* be the length of the coordinate sequence, that is, the number of 1 element in the position matrix. Therefore, the coordinates of the agent's position in a given area at time *t* are (pos_*x*_, pos_*y*_)=(*β*∑*x*_coor_/num, *β*∑*y*_coor_/num), to realize the precise positioning of the agent in a given area.

## 3. Results

To verify the validity of the model, the following experiments are designed: (1) grid cell development experiment, including the effect of the development process of the fringe cell fringe wave and the effect of the development process of the grid cell obtained by the oscillation interference model; (2) place cell development experiment, including the use of BP neural network to simulate the development process of place cells and the relationship between the maturity of place cell populations and the increase in training times; (3) physiological trajectory positioning experiment, using mature cell populations to achieve precise positioning of agent in a given area through an iterative model; (4) map construction experiment, containing the comparison between the position matrix and the discharge activity of the RatSLAM pose cell plate and using the iterative model as the robot platform map construction experiment of the robot positioning system.

### 3.1. Grid Cell Development Experiment

First, the RNNPB is used to simulate the changes in discharge characteristics during the development of stripe cells. Use the self-motion clue information (velocity and direction) in the physiological trajectory of Hafting et al. [3] to obtain the velocity component of the velocity in the corresponding stripe wave direction and use it as the PB bias node input of each stripe wave development unit. The theoretical stripe cell discharge rate during the physiological trajectory is used as a developmental sample. The simulation experiment sets the number of grid cells to be developed as 10, corresponding to the number of stripe cells to be developed as 3×10. Among them, the stripe wave spacing is randomly selected within 10 cm∼70 cm, and the number of hidden layer neurons in each stripe wave development unit is set to 40. The BPTT algorithm and the PB node correction algorithm are used to correct the connection weight of the neural network, and the learning rate of the neural network is set to 0.005.  Figure 9 shows the output change of a stripe wave development unit. It can be seen from the figure that as the number of learning and training times increases, the developed stripe wave gradually approaches the theoretical two-dimensional cos waveform, thereby simulating the changes in discharge characteristics during the development of stripe cells. The given spatial area is a square area of 200 cm*∗*200 cm, the phase of the grid field to be developed is randomly selected in the given spatial area, and the orientation of the grid field is randomly selected within the range of 0°∼360°.  Figure 10 shows the development process of 4 grid cells randomly selected from 10 grid cells. Through the oscillatory interference mechanism, the grid field gradually presents a stable regular hexagonal discharge field in a given space area.

### 3.2. Place Cell Development Experiment

After the grid cells have matured, in a square area of 200 cm*∗*200 cm, the firing rate of the grid cells during the physiological trajectory of Hafting et al. is used as the input of the BP neural network, and the theoretical discharge rate of a single cell at the current position calculated by (5) is output. The number of input nodes of the BP network is 20. During the training process, the learning rate of the BP neural network is set to 0.02, the mean square error cut-off threshold is set to 0.004, and the maximum number of iterations is set to 10. The number of place cells to be developed is set to 50, the center of the discharge field is randomly selected in a given space area, and the place field adjustment factor is set to 1.  Figure 11 shows the effect of cell development in 3 locations randomly selected from 50 locations.  Figure 12 shows the change curve of the number of cells where the maturity reaches 95%.

### 3.3. Iterative Model Positioning Experiment

Set the space area as a 200 cm*∗*200 cm square area, and the coordinate origin is selected in the center of the square area. The conversion ratio *β* of the position matrix to the real environment is set to 1, 20 positioning points are randomly selected in the area, and the operation effect of the iterative model is observed based on the positioning points. Since the number of cells in the mature position mentioned above is 50, the maximum number of iterations of the model should be 50.  Figure 13 shows the effect of position matrix iterations with the anchor point coordinates (9, −10) and (−30, 12).

### 3.4. Physiological Trajectory Positioning Experiment

The physiological trajectory positioning experiment is compared with the positioning performance of the RatSLAM algorithm [36]. In a square area of 10 m*∗*10 m, set Hafting et al.'s rat physiological trajectory [14] to scale up 40 times as the motion trajectory of this experiment, and take 180 points on the trajectory as the points to be located, as shown in Figure 14. The place cell population composed of 50 mature place cells is used to solve the current position of the agent using an iterative model at each positioning point, and the linear distance from the coordinates of the algorithm positioning to the actual coordinates is taken as the positioning error. The distribution of positioning error is shown in Figure 15. The running results show that the average positioning error is 0.676 m in the 180-point positioning process. Compared with the 1.267 m positioning error of the RatSLAM algorithm, the model in this article can detect the position of the rat more accurately. The average number of iterations for 180-point positioning is 35.29. Therefore, due to ensuring the accuracy of the algorithm, the efficiency of the algorithm is high, which verifies the accuracy of the model and the effectiveness of running in a simulation environment.

### 3.5. Positioning Experiments of place Cell Development in Different Stages

In the above experiment, when the number of place cells is constant and the cells mature, the accuracy of positioning in a given space area is solved. Set the number of place cells as 20, 40, 60, 80, and 100, with the space area being still set to a square area of 10 m*∗*10 m. Draw the relationship between the average positioning error size and the number of training times under the above-mentioned types of place cells, as shown in Table 1 (the data in the table retain three decimal places). As the number of training times increases, the average positioning error of the group with more place cells decreases faster, and the average positioning error of the cell group with more place cells after maturity is smaller.

### 3.6. Map Building Experiment

The role of the pose cells in the RatSLAM algorithm is like that of the place cells in the hippocampus. They are all integrating the path to realize the expression of the agent's location in the environment. The position recognition model of the algorithm based on the rat brain hippocampal spatial cell development mechanism replaces RatSLAM pose cells as the positioning part of the bionic map construction algorithm, and the original map construction algorithm part is retained to verify the operation effectiveness of the algorithm in the real physical environment. The indoor dataset of Tian et al. in the literature [37] is selected for verification. The dataset contains the odometer and RGB-D information for the robot to explore 1050 s in an office building with a radius of 35 m. Due to the large space area in the real environment, the conversion ratio *β* of the position matrix to the real environment is set to 23.  Figure 16 shows a comparison between the experimental results of map construction using the RatSLAM algorithm and the experimental results of our location recognition model. The average error between the cognitive maps constructed by these two algorithms is 0.116 m, which verifies the effectiveness of the positioning model in the physical environment.

## 4. Discussion

We propose a positional cognition model based on the developmental mechanism of the hippocampus spatial cells in rats. The RNNPB is used to simulate the development of stripe cells and indirectly simulate the changes in discharge characteristics of grid cells during the development through the oscillation interference of fringe waves. The firing rate of the mature grid cells is used as the information input of the place cells, and the BP neural network is used to simulate the activation firing characteristics of the place cells during the development process. After the place cells are mature, the iterative matrix generated by the place cell population is used for iterative calculation to obtain the location matrix to realize the position recognition of the rat in a given space.

The model in this article is completely based on the physiology of rat brain hippocampal spatial cells. Through spatial cell development experiments, iterative model positioning experiments, and cognitive map construction experiments, it is shown that the model can not only simulate the environmental cognitive mechanism of the hippocampus structure of the rat, but also achieve precise positioning in a given spatial area. The model in this article is position recognition in a given space area, but it fails to realize position recognition in any size space. Generally, the navigation tasks to be performed by mobile robots are carried out in an unknown environment. Therefore, the next research direction is to build a developmental model of spatial cells from the perspective of cognitive mechanism and strive to gradually form and develop the cognitive ability of the environment during the interaction between the robot and the environment. The purpose is to improve the robot's cognitive ability in complex and large-scale space. In summary, the position cognition model based on the rat brain hippocampal spatial cell development mechanism proposed in this paper is of great significance to the research of robot navigation, environmental cognition, and map reconstruction.

## Figures and Tables

**Figure 1:** Map of developmentally activated discharge rates of place and grid cells [16]. (a) Development of place cells recorded in rat hippocampal region CA1. From left to right, the activation firing rate of place cells in rats from postnatal day 16 to postnatal day 29. (b) Development of grid cells recorded in rat medial entorhinal cortex (MEC). The dark blue area above is the firing rate maps of grid cells and the light blue area below is spatial autocorrelograms for grid cells.

**Figure 2:** Schematic diagram of the overall operation mechanism of the model (including grid cell and place cell development model and location cognition model).

**Figure 3:** Wild rendering of grid based on stripe wave oscillation interference model.

**Figure 4:** Grid cell development model structure based on RNNPB.

**Figure 5:** The structure of RNNPB (a) in learning mode and (b) in prediction mode.

**Figure 6:** Structure diagram of place cell development model based on BP neural network.

**Figure 7:** Effect diagram of cell discharge rate at different maturities. From left to right, the effect of cell discharge rate at the position of maturity of 43%, 67%, 89%, and 100%.

**Figure 8:** Schematic diagram of the operation mechanism of the iterative model of mature cells.

**Figure 9:** A schematic diagram of the change of discharge characteristics during the development of a single stripe wave development unit. The green line in each graph represents the theoretical two-dimensional cos wave, and the red line represents the stripe waveform exhibited by the RNNPB through multiple learning.

**Figure 10:** Effect diagram of discharge characteristic changes during grid cell development.

**Figure 11:** Effect diagram of the change of discharge characteristics during the development of place cells. As the number of training times increases, the firing area of the place cell changes from the initial chaotic firing field to the final single-peak firing field, which better simulates the changes in the activation firing during the development of the place cell.

**Figure 12:** The change curve of the number of cells in the position where the maturity reaches 95%. As the number of training times increases, the number of place cells where the maturity reaches 95% gradually increases. In the 4th training, the number of place cells in the 95% maturity increased rapidly from 11 to 43. Moreover, at the end of the 7th training, there were 49 place cells reaching 95% maturity.

**Figure 13:** Running effect of iterative model. The cut-off iterations of the first and second positioning points are 33 and 41, respectively. Through the solution of the iterative model, the position matrix can generate the unimodal activity field of the corresponding position to ensure the accurate positioning of the agent position in a given area. (a) The iterative process of the first locating point. (b) The iterative process of the second locating point.

**Figure 14:** Physiological trajectory and diagram of 180 undetermined sites.

**Figure 15:** Distribution effect diagram of positioning error.

**Figure 16:** The experimental results of RatSLAM positioning algorithm are compared with those of our positioning algorithm. The construction effects of the two cognitive maps are basically the same.

**Table 1:** Data table of mean positioning errors of cell populations in different locations during development.

Number of place cells	Train times						
	1 (m)	2 (m)	3 (m)	4 (m)	5 (m)	6 (m)	7 (m)
20	7.228	7.106	5.723	2.715	2.041	1.808	1.759
40	7.523	7.368	5.452	1.501	0.933	0.874	0.727
60	7.751	7.561	5.085	1.306	0.835	0.691	0.590
80	7.884	7.674	4.632	1.129	0.748	0.508	0.481
100	7.773	7.531	4.003	0.912	0.687	0.474	0.438

## Data Availability

The data used in this study are available from the corresponding author upon request.
